# Procedural Efficiency, Efficacy, and Safety of High-Power, Short-Duration Radiofrequency Ablation Delivered by STSF Catheter for Paroxysmal Atrial Fibrillation

**DOI:** 10.1155/2022/6009275

**Published:** 2022-08-08

**Authors:** Cheng Cheng, Banglong Xu, Jianlong Sheng, Zheng Huang, Fei He, Feng Gao, Xiaochen Wang

**Affiliations:** Department of Cardiology, The Second Hospital of Anhui Medical University, Furong Road 678, Hefei, Anhui 230601, China

## Abstract

**Objectives:**

To investigate the procedural efficiency, efficacy, and safety of high-power, short-term radiofrequency ablation delivered by the SmartTouch Surround Flow (STSF) catheter for paroxysmal atrial fibrillation (AF).

**Methods:**

We retrospectively analyzed a total of 72 patients who were admitted with paroxysmal AF, and who underwent radiofrequency catheter ablation (RFCA) for the first time. Of these patients, 36 cases underwent low-power, long-duration (LPLD, (30–35 W/20–40 s) pulmonary vein isolation (PVI) delivered by an SmartTouch (ST) catheter (control group), and the other 36 cases underwent high-power, short-duration (HPSD, (45–50 W/10–20 s) PVI delivered by a STSF catheter (study group). The baseline data, duration of PVI, procedural time, fluoroscopy time, the rate of first-pass isolation, irrigation perfusion, eschar and steam pop occurrences, intraoperative complications, and the rate of stable sinus rhythm maintenance following a blanking period of three months were analyzed between the two groups.

**Results:**

The isolation time of bilateral PVI and procedural time in the study group were markedly less than in controls (*p* < 0.01). The rate of first-pass isolation in the study group was significantly higher than in the control group (95.8% vs. 84.7%, *p* = 0.023), while the fluid perfusion in the study group was approximately 20% less than that in the control group (767 ± 171 vs. 966 ± 227 ml, *p* < 0.001). We observed no severe complications in any patients. The rate of freedom from AF recurrences following a blanking period of three months showed a tendency to be higher than in controls (93.9% vs. 87.1%, *p* = 0.348).

**Conclusions:**

The HPSD strategy delivered by the STSF catheter was superior to conventional LPLD ablation through the ST catheter with respect to efficiency, acute procedural effectiveness, short-term safety, and the risk of heart failure in patients with paroxysmal AF.

## 1. Introduction

Radiofrequency catheter ablation (RFCA) is an important therapeutic intervention in the management of sinoatrial rhythm control with atrial fibrillation (AF), and has been applied broadly in recent years [1]. Pulmonary vein isolation (PVI) is the cornerstone of therapy for paroxysmal AF [2], and continuous and transmural tissue damage caused by radiofrequency energy for complete PVI is key to preventing the recurrence of AF. Contact force (CF), energy delivery, and ablation time are critical factors with respect to lesion transmurality and uniformity, and catheter stability and the width of lesions determine linear continuity. Many centers have in recent years adopted a traditional low-power, long-duration (LPLD) ablation strategy, and in previous clinical practice at our center, the effect of using an LPLD strategy guided by the ablation index (AI) for PVI was overwhelmingly positive. However, even for skilled operators, the overall procedural time is generally more than two hours, and the procedural efficiency requires improvement. Recent investigations revealed that a high-power, short-term (HPSD) ablation strategy not only shortened ablation time, expanded lesion width, and improved point-to-point connectivity, but also reduced lesion depth and surrounding tissue injury. Additionally, HPSD's procedural efficiency, efficacy, and safety have been demonstrated in numerous clinical studies [3, 4].

The development of ablation catheters has focused on optimizing safety and efficiency in the past decade, and the application of a contact force (CF) pressure sensing catheter is a relatively new and important modality. Therefore, a large number of data from the Symptomatic Paroxysmal Atrial Fibrillation (SMART) AF^5^ study and the Ablation Catheter Study for Atrial Fibrillation (TOCCASTAR) have confirmed the advantage of pressure sensing using short-and long-term outcomes [5–7]. SmartTouch Surround Flow (STSF) is a novel CF-optimized catheter, where its micropore perfusion is increased from a six-hole version in the SmartTouch (ST) catheter to a 56-hole catheter, which greatly induces a better cooling effect of the catheter tip, better energy delivery, better lesion transmurality, and less eschar. This technology also possesses six symmetrical temperature sensors that accurately monitor the temperatures of the catheter and tissue surface in real time. However, the differences between LPLD ablation strategy delivered by ST catheter and HPSD ablation strategy delivered by STSF catheter are limited. Therefore, we herein employed 45–50 W of power with the STSF catheter or 30–35 W of power with an ST catheter for radiofrequency catheter ablation (RFCA) guided by AI in patients with paroxysmal AF. This allowed us to demonstrate procedural efficiency, efficacy, and safety of HPSD as delivered by an STSF catheter.

## 2. Methods

### 2.1. Study Population

In the retrospective single-center study, we analyzed a total of 72 patients who were admitted to the Department of Cardiology of the Second Hospital of Medical University from January 2020 to November 2021 for catheter ablation of paroxysmal AF for the first time, comprising 47 men and 25 women. Of these, 36 patients underwent an LPLD ablation strategy delivered by ST catheter (control group), and the other 36 cases underwent an HPSD ablation strategy delivered by STSF catheter (study group).

Our inclusion criteria were: (1) patients 18–86 years of age with or without symptomatic paroxysmal AF; (2) patients with nonvalvular AF; (3) patients without previous catheter ablation. The exclusion criteria were as follows: (1) patients with valvular or congenital heart disease; (2) a left atrial (LA) anterior posterior diameter >60 mm; (3) a left ventricular ejection fraction (EF) < 40%; (4) an intra-atrial thrombus; (5) acute coronary syndrome; (6) severe renal insufficiency, with an estimated glomerular filtration rate (eGFR) < 30 ml/min/1.73 m^2^; and (7) patients with severe infection, recent surgery, or who experienced cerebrovascular accidents. All of the patients met RFCA indications and signed the informed consent form for RFCA. This study was approved by the local of Research Ethics Committee (YX2022-027), and performed according to the Helsinki Declaration as revised in 2013.

### 2.2. Study Methods

#### 2.2.1. Baseline Data Collection

We collected data on age, sex, height, and weight, as well as patient history of hypertension, diabetes, coronary heart disease, heart failure, stroke, or transient ischemic attack (TIA), and the course of AF. Routine blood chemistry, biochemistry, coagulation tests, and electrocardiography (EKG) examinations were completed prior to the operation; and we assessed patient CHA_2_DS_2_-VASc and HAS-BLED scores [8]. After admission, the patients were treated with anticoagulants (low-molecular-weight heparin or rivaroxaban), and the presence of thromboses was determined by transesophageal echocardiography (TEE). Those individuals who could not tolerate TEE underwent three-dimensional (3D) reconstruction of the left atrium and pulmonary veins (PVs) by multi-slice CT.

#### 2.2.2. Catheter Ablation

All of the patients at our center underwent local anesthesia with lidocaine, and a decapolar catheter (Biosense Webster, CA, USA) was placed within the coronary sinus (CS) via their left subclavian vein or a femoral-vein access. After successful puncture of the atrial septum, heparin (Wanbang Biopharmaceuticals, China) (75–100 u/kg) was injected, and anticoagulation was continued during the operation. The dosage of heparin was adjusted according to the Activated Clotting Time of Whole Blood (ACT) to generate a value between 250 and 300 s. A PentaRay NAV eco High-Density Mapping Catheter (Biosense Webster, CA, USA) was inserted in order to construct an electroanatomic map of the left atrium and PV as guided by a Carto 3D electrophysiological mapping system in the FAM model (Carto3, Version 6, Biosense Webster, CA, USA). All of the patients then underwent point-to-point quantitative circumferential ablation of the pulmonary vein guided by AI. Lesion tags were generated through the VisTag model (Carto VISITAG™ Module, Biosense Webster, CA, USA), and our center tag settings were as follows: a maximal range of catheter movement during ablation of 2.5 mm, a minimal time of catheter stability of 3 s, and a lesion-tag display size of 3–5 mm.

In the power-control mode, the control group underwent an LPLD approach (30–35 W for 20–40 s) delivered by ST catheters (Biosense Webster, CA, USA); and the study group experienced a HPSD approach (45–50 W for 10–20 s) delivered by STSF catheters (Biosense Webster, CA, USA) (Figure 1). Different AI thresholds, ablation times, and power settings in various left atrial sites are shown in Table 1, and we targeted a CF range of 5–20 g. The ST or STSF catheter tip was irrigated by saline at a flow rate of 2 mL/min in the nonablation state; in the ablation state the irrigated flow rate of the ST catheter tip was 16 mL/min (25 mL/min if the power was greater than 30 W), and the irrigated flow rate of the STSF catheter tip was 16 ml/min. Upon completion of PVI, the PentaRay NAV eco high-density mapping catheter was used to verify the PVI (first-pass isolation); if there was an absence of isolation, touch-up ablation was performed until complete PV isolation was achieved.

After the completion of PVI, cardiac electrophysiology was implemented to assess whether there were other arrhythmias. During the procedure, fentanyl citrate (YICHANG HUMANWELL PHARMACEUTICAL CO, LTD, China) (5–15 ml/h·kg) was injected intravenously for continuous analgesia and adjusted according to the pain felt by patients; and blood pressure, heart rate, and blood oxygen saturation were continuously monitored. We observed whether there was eschar or audible steam pop and recorded the ablation time of the left and right PVs, first-pass isolation, fluoroscopy time, total procedural time, and irrigation fluid volume. Postprocedural observations of the puncture site included bleeding, hematoma, pericardial effusion, atrio-esophageal fistula, phrenic nerve injury, and other complications.

#### 2.2.3. Postprocedural Management and Follow-Up

All of the patients were treated with amiodarone (SANOFI, France) or dronedarone (CSPC Pharmaceutical Group Co., Ltd, China) for at least three months postoperatively, with the drugs discontinued if no recurrence was noted or if significant bradycardia developed. The patients were administered warfarin (Shanghai Pharmaceuticals Sine, Shanghai, China) or a new oral anticoagulant (Rivaroxaban, BAYER, Germany, or Dabigatran Etexilate Capsules, Boehringer Ingelheim, Germany) for at least two months, and then evaluated as to whether they were to continue therapy according to the patient's CHA_2_DS_2_-VASc score; and they were placed on a proton-pump inhibitor for at least one month.

All of the patients were advised to follow up at three months and underwent a 12-lead EKG when palpitation symptoms appeared. A 12-lead EKG or Holter monitoring was executed after a 90-day blanking period to observe whether sinus rhythm was achieved or whether bradycardia arrhythmia remained.

#### 2.2.4. Statistical Analysis

We employed SPSS 20.0 (IBM Corp., Armonk, NY, USA) for all statistical analyses. The measurement data were expressed as mean ± SD (fluoroscopy time was expressed in quartiles), and the counting data were expressed as frequencies and percentages (*n* (%)). We used a *t*-test or chi-squared test for comparisons of measurement data or counting data between the two groups, and a Mann–Whitney *U* test for non-normally distributed measurement data. *p* < 0.05 was considered to be statistically significant.

## 3. Results

### 3.1. Baseline Characteristics

A total of 72 patients (61.0 ± 11.1 years of age, 65.3% male) comprised this study, with 36 cases in each of the control and study groups. There were no significant differences between groups with regard to age, sex, or body mass index (BMI); onset time of AF; or patient history of hypertension, diabetes, coronary heart disease, heart failure, or stroke/TIA; nor in eGFR, left ventricular (LV) and LA diameters, EF, or CHA_2_DS_2_-VASc score, and HAS-BLED score (Table 2).

### 3.2. Procedural Parameters

Of the 72 patients, one manifested a left pulmonary vein trunk. In the control group, one patient underwent LA posterior wall linear ablation because LA matrix mapping showed a strip-shaped, low-voltage area of the LA posterior wall. Because AF was induced by programmed atrial stimulation in this patient, we executed LA anterior wall linear + mitral isthmus linear + tricuspid isthmus linear ablation, and a double-block was attained in this patient. In one patient in the study group whose AF originated from the superior vena cava (SVC), we defined the function of the sinoatrial node by an activation map under sinus rhythm, and a 3D distribution of the right phrenic nerve was defined by a pacing map; segmental RFCA was then implemented for SVC isolation. In the study group, one patient underwent LA roof linear + mitral isthmus linear ablation due to atrial programmed stimulation, and a double-block was also attained. The other patient in the study group exhibited induced atrioventricular nodal reentrant tachycardia (AVNRT) and underwent modification therapy of the slowed electrical pathway.

Regarding procedural efficiency, the RF times for PVI of left and right veins in the study group were 32.1 ± 7.0 min and 29 ± 7.0 min, respectively, which were significantly less than in the control group (PVI of left veins, 41.3 ± 6.2 min; PVI of right veins, 33.1 ± 4.5 min, *p* < 0.01). The total procedural time in the study group was also significantly less than that in the control group (111.8 ± 36.1 min vs. 145.4 ± 34.3 min, respectively, *p* < 0.001), but the fluoroscopy time showed no difference between groups (Table 3).

Successful PVI was completely achieved in all patients. The rate of first-pass isolation in the study group was 95.8%, while that of the control group was 84.7% (*p* = 0.023). We observed a marked reduction in the study group in the total irrigation perfusion volume by approximately 20% (767 ± 171 ml vs. 966 ± 227 ml, *p* < 0.001, respectively) (Table 3).

### 3.3. Follow-Up

Clinical follow-up data were available for 33 of 36 (91.7%) patients from the study group and 31 of 36 (86.1%) from the control group at the three-month follow-up. Thirty-one of 33 patients (93.9%) were free of AF recurrence following a blanking period of three months in the study group, whereas the proportion was 27 of 31 (87.1%) in the control group (not significant (NS); *p*=0.348).

### 3.4. Complications

There was no eschar generated in either group during the procedure, and three audible steam pops occurred during ablation in the study groups, with two in the control group. Neither steam pop led to pericardial effusion. In the control group, one patient experienced acute heart failure and one patient experienced acute pancreatitis and diabetic ketoacidosis after ablation. In the study group, one patient manifested bradycardia, but no permanent pacemaker was implanted after the procedure; and one patient exhibited a hematoma at the puncture point of the left shoulder that was associated with the puncture. We observed no atrio-esophageal fistula, SVC stenosis, phrenic nerve injury, or sinoatrial nodal injury in the perioperative period in any patient.

## 4. Discussion

The present study revealed that the HPSD ablation delivered by an STSF catheter not only conveyed distinct advantages in procedural efficiency, acute success, and short-term safety, but also showed a tendency for a higher rate of stable sinus rhythm following three months in the treatment of paroxysmal AF. First, compared with LPLD ablation delivered by an ST catheter, the RF and procedural times for HPSD ablation delivered by the STSF catheter were significantly shortened, which greatly enhanced overall procedural efficiency. Second, the rate of first-pass isolation of HPSD ablation delivered by the STSF catheter was 13.1% higher than that with LPLD ablation delivered by the ST catheter, which ameliorated the acute achievement of PVI. Third, the irrigated fluid volume of HPSD ablation delivered by the STSF catheter was diminished by approximately 20%, which reduced the risk of heart failure caused by volume overload, and HPSD did not elevate procedural risk or the incidence of complications.

Although we have observed an annual increase in the prevalence and incidence rates of AF as China's population ages, the efficacy and safety of traditional antiarrhythmic drugs are currently unsatisfactory. Moreover, while numerous guidelines recommend catheter ablation as the first-line therapy for paroxysmal AF [1, 9], how to improve procedural efficiency and safety and promote short- and long-term success rates remain constant concerns. The continuous and transmural nature of ablation lesions exerts a direct influence on recurrence rate, which is the key to circumferential PVI. Catheter stability, RF power and duration, CF, and temperature of the catheter tip are essential parameters of the lesion size and transmurality, and AI modules can thus be exploited to calculate and quantify the RF parameters and be used to accurately evaluate each ablation point so as to improve procedural success rates [10]. Administrators of one multicenter study have suggested that the rate of one-year's relief from AF recurrences in patients who underwent RFCA guided by AI was 91% with respect to paroxysmal AF [11]. Moreover, since 2019, the rates at our center for one-year relief from recurrences of paroxysmal and persistent AF have been 92.7% and 73.9%, respectively (unpublished data). However, in cases of ablation difficulties, it is necessary to explore more efficient ablation strategies.

High-power (HP) ablation comprises one of the most studied clinical modalities. HPSD ablation enhances resistive heating by increasing RF power so as to achieve wider and more transmural lesions, while it also weakens conductive heating by shortening the ablation time and diminishing the depth of the lesions to avoid injury to the surrounding tissues [12]. Some studies conducted *in vivo* have shown that HPSD ablation increased the width of the lesions and led to better continuity between points and because of the shorter ablation time at a single point, the procedural time was commensurately shortened [13–15]. Although complications such as steam pop, eschar at the catheter tip, and perforation of the left atrium may occur during HP ablation, the STSF catheter, in theory, reduces these complications by optimizing irrigation at the catheter tip. The STSF catheter possesses 56 irrigation holes and allows precise temperature sensing to homogeneously cool the catheter tip, which avoids gasification of water in the tissues and the interruption of ablation caused by overheating. In addition, optimal cooling of the ablation electrode provides a more efficient RF delivery and generates transmural lesions more easily [16].

In the present study, we retrospectively analyzed patients with paroxysmal AF who underwent RFCA for the first time at our center between January of 2020 and November of 2021. The ST catheter was employed for LPLD ablation at a power of 30–35 W, and 30 W was applied for 20–25 s during posterior wall ablation due to possible esophageal injury. The STSF catheter was used for HPSD ablation with a power of 45–50 W, while 45 W was applied for 10–15 s during posterior wall ablation. Our results revealed that the rate of first-pass isolation in the HPSD group with the STSF catheter was 95.8%, which was 13.1% higher than that in the LPLD group with the ST catheter (*p* = 0.023), similar to the findings of Phlips et al. [17]. We hypothesized that the HPSD approach with an STSF catheter improved acute success, and a large number of clinical studies have further confirmed the short-term efficacy outcomes of the HPSD method [18–20]. While numerous recent studies have shown that HPSD ablation resulted in higher first-pass isolation and lower PV reconnection [4, 21], whether the HPSD method reduces the long-term recurrence rate of AF is still controversial. A recent meta-analysis showed that RFCA using HPSD effectively reduced the risk of recurrent AF (RR = 0.72; 95% CI = 0.54 to 0.96; *p* = 0.02), but not of atrial flutter (AFL) or atrial tachyarrhythmia (AT) [4]; and a second meta-analysis revealed that the HPSD strategy did not lessen relief from atrial tachyarrhythmia at 12-month follow-up [22]. Moreover, a retrospective study by Baher et al. depicted a similarity in AF recurrence rates between HPSD and LPLD ablation at a mean follow-up period of 2.5 years (42% vs. 41%, respectively, *p* = 0.571) [23]. It is worth noting that the STSF catheter is superior to the ST catheter in ablation efficacy [24, 25], and that PVI by the STSF catheter reduces the rate of early reconnections of the left PV [26]. Likewise, there was a trend toward improved efficacy of the STSF ablation catheter compared to the ST device in the Kaplan–Meier estimation of 12-month arrhythmia-free survival (NS, *p* = 0.18) [27]. In the present study, the HPSD strategy delivered by the STSF catheter not only improved the rate of first-pass isolation but also showed a tendency for a higher rate of stable sinus rhythm following a blanking period of three months (93.9% vs. 87.1%, *p* = 0.348, respectively, NS). Bunch et al. [28] analyzed the 3-year prognosis of patients undergoing HPSD ablation and those with conventional ablation, and also found no significant difference in the 3-year AF recurrence rate between the two ablation strategies (26.5% vs. 30.7%; *p* = 0.23), which was similar to the prognostic results in this study. Clinical studies with larger sample sizes and longer follow-up times are needed in the future to clarify these potential differences in rates.

Many recent studies have revealed that RFCA using HPSD greatly improves procedural efficiency [18, 23, 29]. In the present study, we established that HPSD ablation delivered by STSF catheter significantly shortened ablation time, thus greatly improving procedural efficiency, which is consistent with the research results of Dhillon et al. [30]. Our results also showed that the PVI times of the left and right PVs with the HPSD method and using the STSF catheter were 32.1 ± 7.0 min and 29 ± 7.0 min, respectively, which were notably shorter than times in the LPLD group (41.3 ± 6.2 min and 33.1 ± 4.5 min, respectively). Importantly, the total procedural time was reduced to less than 120 min. Because the width of the lesions in HPSD ablation was large, lesion continuity was nevertheless assured even when ablation points were few. The ablation time at a single point was greatly shortened, and the total procedural time was also abbreviated accordingly.

The short ablation time at every point was also more conducive to the stability of catheter manipulation. In addition, we found that the fluoroscopy time for HPSD with the STSF catheter was slightly but not significantly reduced; this might portend an association with a clearer display of potential signals during the procedure [31].

It is indisputable that although an HPSD strategy improves overall procedural efficiency and efficacy, it also poses some safety issues. The control of CF and RF duration comprises the critical determinant in complication prevention. As CF increases, the risk of myocardial perforation increases, and excessive CF also affects the flow rate of saline irrigation at the catheter tip, elevating the risk of eschar. Insufficient RF time causes inadequate ablation and results in nontransmural lesions, while excessive ablation may conversely lead to steam pop, pericardial effusion, esophageal and phrenic nerve injury, thrombosis, and stroke. The unique 56-hole irrigated cooling design reduces the occurrence of steam pop and eschar [24], and we observed acute safety with HPSD ablation as delivered by the STSF catheter in the present study. Although we noted no pericardial tamponade, atrio-esophageal fistula, or pulmonary vein stenosis in either the LPLD or HPSD groups we did observe steam pop in three cases of the HPSD group, but this was not significantly different from the LPLD group. Qu et al. [32] showed that the occurrence of steam pop was significantly related to HP under RFCA intervention, which was different from our study. The reason may be related to the improved thermostability of the STSF catheter after optimization in this study.

Continuous high-flow irrigation during procedures may precipitate congestive heart failure (CHF), and thus fluid management is particularly important for patients with pre-existing CHF. In one study, the researchers demonstrated that the irrigation fluid volume using the STSF catheter during PVI was 51.7% less than that with the ST catheter [27]. Furthermore, our study similarly showed that irrigation fluid volume using the STSF catheter was dramatically reduced, and we also noted no incidence of heart failure after the procedure. Thus, patients who have previously experienced CHF may benefit more from the use of the STSF catheter.

Although the effectiveness and safety of RFCA using HPSD have been disclosed, the levels of power that afford the best efficacy and safety—and the upper limit of power—remain ambiguous. Since our center had no prior experience in high-power ablation, we adopted RFCA with a power of 45–50 W and a duration of 10–20 s. There exist very few studies on very-high-power, short-duration (vHPSD) ablation. One center used 70 W for very high-power or 30–40 W for conventional power for PVI in paroxysmal AF, and these authors found that the vHPSD approach exhibited markedly fewer AF recurrences after one year—with a satisfactory safety profile [33]. Moreover, some studies comprising a 90-W ablation mode provided safe and efficient PVI [34, 35]. We will therefore further explore higher-power ablation in the future to observe its effectiveness and safety.

### 4.1. Limitations

The current study entailed some limitations. First, this was a retrospective study of a single-center experience, with a limited number of patients enrolled. Additional studies of larger sample sizes and that encompass multiple centers are therefore required to confirm these findings. Second, the follow-up period was limited to three months, and a follow-up based upon using a 12-lead EKG or Holter-monitor examination may have underestimated the actual incidence of atrial arrhythmia. Thus, additional studies with long-term follow-up and more robust arrhythmia monitoring are necessary to demonstrate efficacy and safety. Third, since this study was focused on efficacy in first-time AF-ablation patients, we will in the future examine patients undergoing repeated ablations.

## 5. Conclusions

This study suggests that the HPSD strategy delivered by an STSF catheter in patients with paroxysmal AF is more efficient and that it exhibits a higher rate of first-pass isolation, necessitating a smaller volume of fluid irrigation, and satisfies safety aspects. However, long-term efficacy and safety need to be further evaluated in the future.

## Figures and Tables

**Figure 1:** PVI in paroxysmal AF. (a) LPLD (40 W/31 s, AI 500) ablation delivered by an ST catheter. (b) HPSD (50 W/19 s, AI 490) ablation delivered by an STSF catheter.

**Table 1:** RF power, AI thresholds, and RF time per lesions in different left atrial sites.

	Group	Anterior	Ridge	Roof	Inferior	Posterior
RF power	Control	35 W	35 W	35 W	35 W	30 W
	Study	50 W	50 W	50 W	50 W	45 W

AI	Control	450–480	480–500	400–450	400–450	380–420
	Study	450–480	480–500	400–450	400–450	380–420

RF time per lesions	Control	30–40 s	35–40 s	25–35 s	25–35 s	20–25 s
	Study	15–20 s	15–20 s	10–20 s	10–20 s	10–15 s

RF, radiofrequency; AI, ablation index.

**Table 2:** Baseline demographic and patient characteristics.

Characteristics	Control group (*n* = 36)	Study group (*n* = 36)	*p* value
Sex (male/female)	20/16	27/9	0.083
Age (years)	63.11 ± 9.96	58.92 ± 11.92	0.110
BMI (kg/m^2^)	25.38 ± 3.24	24.11 ± 2.98	0.089
Hypertension (*n* (%))	18 (50.0)	20 (55.6)	0.637
Diabetes (*n* (%))	7 (19.4)	6 (16.7)	0.759
Coronary heart disease (*n* (%))	11 (30.6)	6 (16.7)	0.165
Heart failure (*n* (%))	3 (8.3)	1 (2.8)	0.303
Stroke/TIA (*n* (%))	4 (11.1)	2 (5.6)	0.394
Mean AF duration (months)	28.31 ± 31.46	35.50 ± 36.38	0.716
CHA_2_DS_2_-VASC	2.31 ± 1.95	1.69 ± 1.49	0.191
HAS-BLED	0.64 ± 0.59	0.44 ± 0.61	0.130
eGFR (ml/min/1.73 m^2^)	89.48 ± 20.71	91.66 ± 26.94	0.165
LA diameter (mm)	38.08 ± 6.40	38.19 ± 6.46	0.942
LV diameter (mm)	45.31 ± 5.06	47.31 ± 4.62	0.084
LV EF (%)	61.53 ± 4.07	63.04 ± 4.40	0.136

Data are expressed as mean ± SD or *n* (%). BMI, body mass index; TIA, transient ischemic attack; AF, atrial fibrillation; eGFR, estimated glomerular filtration rate; LV, left ventricular; EF, ejection fraction.

**Table 3:** Procedural characteristics and freedom from AF recurrences following a blanking period of three months.

Characteristics	Control group (*n* = 36)	Study group (*n* = 36)	*p* value
Left PVI time (min)	41.3 ± 6.2	32.1 ± 7.0	<0.001
Right PVI time (min)	33.1 ± 4.5	29.1 ± 7.0	0.007
Procedural time (min)	145.4 ± 34.3	111.8 ± 36.1	<0.001
Fluoroscopy time (min)	4.5 (4.0–5.0)	4.0 (3.25–5.0)	0.129
First pass isolation *n* (%)	61/72 (84.7)	69/72 (95.8)	0.023
Irrigation fluid volume (mL)	966 ± 227	767 ± 171	<0.001
Steam pop (*n* (%))	2 (5.6)	3 (8.3)	0.643
Freedom from AF recurrences (*n* (%))	31/33 (93.9)	27/31 (87.1)	0.348

Data are expressed as the mean ± SD or *n* (%) (fluoroscopy time was expressed in quartiles). PVI, pulmonary vein isolation; AF, atrial fibrillation.

## Data Availability

The labeled dataset used to support the findings of this study are available from the corresponding author upon request.
